# Failure analysis in predictive maintenance: Belt drive diagnostics with expert systems and Taguchi method for unconventional vibration features

**DOI:** 10.1016/j.heliyon.2024.e34202

**Published:** 2024-07-06

**Authors:** Ahmed Adnan Shandookh, Ahmed Ali Farhan Ogaili, Luttfi A. Al-Haddad

**Affiliations:** a Mechanical Engineering Department, University of Technology- Iraq, Baghdad, Iraq; b Mechanical Engineering Department, University of Mustansiriyah, Baghdad, Iraq; c Training and Workshops Center, University of Technology- Iraq, Baghdad, Iraq

**Keywords:** Belt drive, Random forest, Taguchi method, Predictive maintenance, Failure analysis

## Abstract

Predictive maintenance to avoid fatigue and failure enhances the reliability of mechanics, herewith, this paper explores vibrational time-domain data in advancing fault diagnosis of predictive maintenance. This study leveraged a belt-drive system with the properties: operating rotational speeds of 500–2000 RPM, belt pretensions at 70 and 150 N, and three operational cases of healthy, faulty and unbalanced, which leads to 12 studied cases. In this analysis, two one-axis piezoelectric accelerometers were utilized to capture vibration signals near the driver and pulley. Five advanced statistics were calculated during signal processing, namely Variance, Mean Absolute Deviation (MAD), Zero Crossing Rate (ZCR), Autocorrelation Coefficient, and the signal's Energy. The Taguchi method was used to test the five selected features on the basis of Signal-to-Noise (S/N) ratio. For classifications, an expert system was used based on artificial intelligence where a Random Forest (RF) model was trained on untraditional parameters for optimizing the accuracy. The resulted 0.990 and 0.999, accuracy and AUC, demonstrate the RF model's high dependability. Evidently, the methodology highlights the features potential when progressed into expert systems, which advances predictive maintenance strategies for belt-drive systems.

## 1 Introduction

### 1.1 General overview

Generally speaking, failure prevention, fatigue avoiding, and predictive maintenance stand as ones of the major advancements when it comes to maintenance strategies of modern mechanical systems [1,2], specifically in belt drive mechanical systems [3,4]. This prediction-based approach acts as a main pillar in fault prevention to avoid system failures to ensure high operational accuracy and safety [5,6]. Belt drives, integrally related to numerous industrial machines, demand constant monitoring due to their critical role and susceptibility to various forms of wear and deterioration [7,8]. The essence of predictive maintenance lies in its ability to forecast potential failures and facilitate timely interventions where this foresight primarily hinges on the analysis of key indicators that reflect the system's health [9,10]. Among these methodologies lies vibration analysis which is a widely recognized and powerful technique of timely fault detection and prevention [[11], [12], [13], [14]]. It leverages the vibrational signatures of machinery to identify abnormalities and potential wear, unbalance, or damage, long before they escalate into major failures [15,16].

In belt drive mechanical systems, vibrational signal patterns can reveal a multitude of conditions, starting with belt misalignment and tension irregularities to more subtle indications of wear or impending breakdown [17]. The ability to accurately interpret these vibrations is crucial for maintaining the reliability and longevity of these systems. This necessitates not only an understanding of the mechanical aspects but also an adeptness in the analytical techniques that can decode the complexities hidden in vibrational data [18]. Moreover, as industries increasingly lean on data-driven decision-making nowadays, the integration of advanced analytical methods with traditional mechanical systems opens new avenues in predictive maintenance [[19], [20], [21]]. This synergy is where this paper aims to contribute, bridging the gap between mechanical expertise and data analytics to enhance the reliability of belt-drive systems.

### 1.2 Literature survey

Recent advancements in predictive maintenance for belt drive systems have been significantly influenced by previously published innovative methods to data analysis and decision-making frameworks. For instance, Liu et al. (2019) proposed an integrated maintenance decision-making methodology for belt conveyor idlers where varying thresholds were used based on real-time operational conditions and reliability estimation results with a notable deviation from traditional constant threshold-based diagnostics [22]. Similarly, Ouerghemmi et al. (2023) introduced a dynamic model for V-belt transmission systems by the employment of spectral analysis techniques like Motor Current Signature Analysis (MCSA) and Extended Park Vector Approach (EPVA) to detect belt faults and the results demonstrated EPVA's higher sensitivity to defects [23]. Additionally, Pollak et al. (2021) emphasized the significance of anomaly detection based on vibrations for predictive maintenance in Industry 4.0 platforms that presented a method that aids in the estimation of the remaining service life of belt drive components [24].

To continue exploring other conducted works, Rumin et al. (2023) described the use of machine learning algorithms in conjunction with analytical calculations to predict belt flip over in conveyor belts in the field of information technology to prevent failures in modern industrial setups [25]. Furthermore, Fehsenfeld et al. (2023) has tackled the challenge of limited fault data availability by proposing a multi-source domain adaptation procedure that integrates synthetic fault data generation into cross-domain classifier training, specifically for diagnosing faulty pretensioning of belt drives [26]. Lastly investigated, Baqer et al. (2023) has developed an intelligent system for detecting belt drive contamination status using vibration signal analysis and an Artificial Neural Network (ANN), showcasing the efficacy of time-domain signal analysis in identifying various operational conditions that stated the potential of time-domain signals [27]. Table 1 elaborates on recent belt-drive system diagnostical methodologies it terms of different specifications and approaches.

**Table 1:** Recent state-of-the-art on belt driven systems’ diagnostical techniques.

Ref.	Application	Type of Signal	Use of Signal Processing	Statistical Features	Use of Expert System
[24]	Predictive Maintenance	Vibration	Anomaly detection based on vibration data	N/A	Not specified
[27]	Contamination Status Detection	Vibration	Time-domain signal analysis; feature extraction using Matlab Simulink	RMS, Kurtosis, Skewness	ANN
[28]	Fault Diagnosis and Classification	Vibration	Wavelet enveloped power spectrum	Time features extracted from wavelet transform	SVM
[29]	Condition and Behavior Diagnostics	Vibration	Numerical-experimental procedure; Finite element method for diagnostics	N/A	No, uses numerical-experimental procedures
[30]	Fault Diagnosis under Non-stationary Conditions	N/A	Theoretical evaluation and industrial testing	N/A	Not specified, ad hoc signal-based methods
[31]	Fault Diagnosis	Vibration	Comparison of new and existing diagnostic methods through experiments	N/A	No, focuses on vibration analysis methods

### 1.3 Originality and significance

While existing studies in the field of predictive maintenance for belt-drive systems have progressed heavily, certain limitations continue to appear. Relying on static threshold-based traditional feature analysis decision-making is a common drawback, which may not adequately account for the dynamic nature of operational conditions [22]. Adding up, methods like the earlier discussed EPVA, although adequately effective, often require extensive data for accurate fault detection, limiting their applicability in specific situations with limited data acquisition [23]. Many of these studies also tend to focus on specific aspects of belt-drive systems, such as fault detection or tension irregularities, without a holistic approach to full system health monitoring for proactive decision-making. The integration of advanced data analytics and machine learning techniques in these studies is apparently in its early stages, with limited exploration of their full potential in the enhancement of predictive maintenance approaches [32]. To address these research gaps, this paper introduces several novel.

• A Comprehensive analysis across diverse operational states of a belt drive system of varying speeds, pretension levels, and conditions (healthy, faulty, unbalanced).
• The utilization of advanced statistical features from vibration data for a deeper analysis, including Variance, MAD, ZCR, Autocorrelation, and Energy.
• The use of Taguchi method for the purpose of demonstrating the importance of each of the selected five features.
• The application of an expert system RF method with specific selected parameters to enhance the classification accuracy.
• Opening doorways for future predictive maintenance strategies that employ a novel decision-making approach with a depend on advanced statistics.

## 2 Experimental approach and data acquisition

### 2.1 Test rig and failure methodology

This research paper has utilized an experimental data from a previously published study that focused on vibration analysis for condition monitoring of belt-drive mechanical systems. The collected datasets, as outlined in the study by Khalifa et al. (2023) [33], contains a wide range of operational states, providing the rich foundation for the analysis and subsequent RF-based machine learning application when progressed into classification purposes.

To understand the experimental approach of this study, it is important to point out that the G.U·N.T machinery setup for diagnostics (PT 500.14) was thoroughly used in the cited reference of experimental methodology. The conducted experiment, along with the test rig of the belt-drive mechanism, is depicted in Fig. 1. The system is composed of a PT 500 base unit, including an electric motor, a shaft, and two bearing blocks as shown in the same Figure. The motor's speed (*N*) is controllably varied using a speed controller, offering a wide range of operational rotational velocities. While in this research, two specific operational speeds were chosen, namely 500 RPM for low dynamic response and 2000 RPM for high dynamic spectrum. In addition to that, to understand the connection methodology, an elastic coupling connects the motor to the shaft, facilitating good alignment and highly operated flexibility, while ball bearing-supported blocks stabilize the shaft. Moreover, Central to the setup is the pre-tensioned V-belt, an SPZ type with the following measurements: 912 mm in length and 10 mm in width, linking a small driver pulley and a larger driven pulley for the belt-drive mechanical system. This belt is a main component for power transmission to the driven pulley, with a diameter of 125 mm. The belt's tension (*T*) was adjustable with desired levels, for this experimental approach, two distinct levels were specified, 70 and 150 N, respectively. Again, these values were chosen to make sure that both high and low spectral dynamic responses are studied adequately.

**Fig. 1:** G.U·N.T Machinery diagnostic system setup [33].

For the type of utilized accelerometers, two IMI 603C01 piezoelectric sensors [34,35], that capture the vibrational signals of one axis, were positioned onto the blocks of the bearings in the test rig. One of the accelerometers was affixed onto the bearing of the shaft that holds the driven pulley, and the other one onto the bearing holder of the driver pulley, respectively. After amplification, these signals were digitized using a USB data acquisition card (BMCM) and processed through LabVIEW for analysis [36] where the data were saved directly into a measurement file to hold the time-domain vibrational signal patterns.

To systematically analyze fatigue and failure within the belt drive system, the study conducted controlled tests that simulate operational stress and wear over extended periods. These tests are designed to incrementally increase the load and operational tempo. In addition to a close monitoring of the onset of wear and eventual failure. For that, and for the purpose of determining he different operational states, the experiments explored vibration signal characteristics under the varying different conditions: two belt tension levels, healthy and faulty operational belts, and mass adding for the purpose of creating intentional imbalances. To further look into the types of how these faults were induced, the three states of studied cases are presented in Fig. 2.

**Fig. 2:** Fatigue and failure introducing: experimental fault setup [33].

This dataset, with its diversity and depth, serves as an ideal platform for exploring the utilized RF model in predictive maintenance. By encompassing a wide range of operational states, the data enables a detailed understanding of vibrational behaviors and dynamic responses under different states and wider spectrum analysis, setting the groundwork for the subsequent analysis and model development in this work. Following up in the next subsection, the advanced features are discussed.

### 2.2 Advanced feature extraction-testing strategy

Novel and unconventional feature selection methodologies are now emerging in many state-of-the-art fields of interest [[37], [38], [39]]. Following up to the current investigation along with the experimental methodology and data acquisition, the extraction of statistical characteristics from the vibrational data takes place. In order to determine the dynamic behavior of the belt-drive system which operates under variant rotational, forced, and unbalanced states, the following statistics are employed. An overview of the aforementioned features in addition to their mathematical expression is enlisted in Table 2.

**Table 2:** Advanced statistical features employed in the current approach.

Feature	Expression
Variance	$\text{Var}\;\left(X\right)=\frac{1}{N}\sum_{i=1}^{N}\;{\left(x_{i}-\mu \right)}^{2}$
Mean Absolute Deviation (MAD)	$\text{MAD}=\frac{1}{N}\sum_{i=1}^{N}\;\left|x_{i}-\mu \right|$
Zero Crossing Rate (ZCR)	$\text{ZCR}=\frac{1}{N-1}\sum_{i=1}^{N-1}\;1\left(s\left[i\right]\cdot s\left[i+1\right]<0\right)$
Autocorrelation Coefficient R(τ)	$R\left(\tau \right)=\frac{1}{N}\sum_{i=1}^{N-\tau }\;\left(x\left[i\right]-\mu \right)\left(x\left[i+\tau \right]-\mu \right)$
Energy of the Signal (E)	$E=\sum_{n=-\infty }^{\infty }\;|x\left[n\right]{|}^{2}$

As stated earlier in Table 1, five specific statistical features are employed. Firstly, the variance that represents the dispersion of the signal from its average mean, reflects the variability that occurs in the adopted vibration datasets [40]. This feature is quite useful in identifying changes and shifts of operational states and conditions leading to deviations from natural and normal patterns [41,42]. The Mean Absolute Deviation (MAD) on the other hand, is a secondary measure of dispersion that provides clear indication of the average magnitude in the vibration samples when deviating from the average mean value of the same signal [43]. MAD is less influenced by the peaks and extreme values, and hence, offers higher effectiveness in understanding variability when compared with the variance. Proceeding further, the Zero Crossing Rate (ZCR) is a key feature and indication of the frequency spectrum with which the signal changes from positive to negative or the opposite [44]. The ZCR feature is quite instrumental in identifying the high-frequency components presence which are highly indicative of mechanical faults or irregularities. Adding up, Autocorrelation Coefficient R(τ) would provide good insights into the similarity of a signal with its delayed version over different time lags τ. This feature is a key instrument in revealing the repetitive or periodic nature of the vibrational datasets, which is crucial for fault diagnosis in rotating machinery [45]. Lastly, the sum of the squared magnitude of the vibration signals is called the Energy of the signal (E) which encapsulates the total energy present in the vibration [46]. It is a pivotal feature for assessing the overall intensity and power of the vibrational activity. In this study, five features were calculated for each of the accelerometers, and hence, 10 statistical features for each case are calculated for classification purposes. The extraction of these features from the vibrational data lays the groundwork for the subsequent machine learning analysis. These features will enable capturing wide ranges of vibration signal datasets which will facilitate detailed understanding of the belt-drive system as progressing into the proposed machine learning model.

Continuedly, the study employs the Taguchi method to optimize feature selection for the predictive maintenance model [47,48]. The methodology involves a series of controlled experiments based on an orthogonal array (OA) that systematically tests combinations of features at defined levels. Each experimental setup's performance is quantified using the Signal-to-Noise (S/N) ratio, specifically the “larger is better” type given by the equation below:

$$\text{SN}=-10\;\log\frac{1}{n}\sum_{i=1}^{N}\;\frac{1}{y^{2}}$$

Where *y* represents the performance metric (e.g., accuracy) and *n* denotes the number of trials.

## 3 Artificial intelligence-based expert system

### 3.1 Random forest algorithm

Expert systems are one of the cornerstones to artificial intelligence which harness rule-based reasoning to emulate human decision-making processes in complex engineering tasks. Artificial intelligence-based methodologies have recently spanned a wide range of mechanical engineering applications [[49], [50], [51], [52], [53], [54], [55]]. In order to guarantee robust and effective vibrational data analyzing for classification purposes, this study implemented the application of Random Forest algorithm for the proposed experimental belt-drive system. RF is an ensemble learning methodology that shines in handling extremely complicated classification problems which involve multiple features in addition to variant operational experimental states [56,57]. The decision trees are the core heart of the RF algorithms, where each one of these trees are constructed depending on a specific subset of data. While constructing these trees, a precise criteria is followed, to determine the best split of each node to make sure each segment of the data is chosen in the most effective pattern. Minimizing the sum of the squared differences from the mean in the two nodes created by the split, is the best criteria to acquire the best split in each potential decision tree. Equation below gives insights into the split methodology, adopted in this study and mathematically presented as [58,59]:

$$Split={\mathrm{argmin}}_{j,t}\left[{\mathrm{Min}}_{Left\;Nodes}\sum {\left(Value-mean\right)}^{2}+{\mathrm{Min}}_{Right\;Nodes}\sum {\left(Value-mean\right)}^{2}\right]$$

where *j* is a specific feature over which the split is made and the threshold value for splitting the data is presented as *t*. Each tree in the Random Forest makes an independent decision or classification based on the input features. The final classification decision of the Random Forest model is then made by aggregating the decisions of all the individual trees, typically using majority voting for classification tasks. This ensemble approach not only improves the predictive accuracy but also mitigates the risk of overfitting, a common challenge in decision tree models. Applying the Random Forest model to the vibration data involves training the model on a labeled dataset, where each data point is characterized by the extracted statistical features and associated with a specific operational state (healthy, faulty, or unbalanced). The trained model is then used to classify new, unseen data, predicting the operational state based on the vibrational characteristics. Fig. 3 illustrates the general approach of the tree creation in the utilized random forest algorithm. Table 3 lists the key parameters utilized in configuring the Random Forest model for this study. The number of trees is set at 100, a value that offers a balanced compromise between model accuracy and computational efficiency. In general, an increase in the number of trees improves the efficacy and stability of the model; however, it also imposes a greater computational load. Consequently, the proposed 100 trees will indicate a robust manageability in the structure of the random forest. The square root of the total number of all features is used to determine which indicators are used at each level of the tree classifier. This will guarantee good leveling diversity in the classifier through the incorporation of different features at each node, eliminating overfitting. The minimal dividing subset size is set at 2, dictating the profundity of every tree in the forest. This will enable the model to acquire comprehensive insights of data patterns and hence, avoiding overfitting once again. These enhanced parameters will further advance the method's capacity for higher accuracy results to indicate the vibrational-dependent classification methodology in the belt-drive system. Hence, this optimization guarantees precise forecasts of the diverse operational states.

**Fig. 3:** Random forest tree variations [60].

**Table 3:** Random forest parameters.

Parameter	Value
No. of trees	100
No. of attributes considered at each split	3
Do not split subsets smaller than	1

### 3.2 Performance assessment and evaluation

Accuracy denotes the frequency with which the classifier predicts the class label with precision, it is determined by dividing the count of accurate predictions by the overall count of predictions. In a more detailed form, considering a confusion matrix with True Positives (TP), True Negatives (TN), False Positives (FP), and False Negatives (FN). Moreover, Area Under the ROC Curve (AUC) is a performance measurement for classification problems at various threshold settings. The ROC is a probability curve, and AUC represents the degree or measure of separability. It tells how much the model is capable of distinguishing between classes. Higher the AUC, better the model is at predicting 0s as 0s and 1s as 1s. An AUC score of 0.5 suggests no discrimination (i.e., random guessing), and 1 represents perfect discrimination. It is calculated such that *n* is the number of points on the ROC curve. $x_{i+1}\;\text{and}\;x_{i}$ are consecutive values of False Positive Rate (FPR). $y_{i}\;\text{and}\;y_{i+1}$ are the corresponding values of True Positive Rate (TPR). AUC does not have a simple equation like Accuracy, as it involves plotting a ROC curve and then calculating the area under this curve. The equations are provided in Table 4 below.

**Table 4:** Utilized advanced statistical features.

Feature	Expression
Accuracy (CA)	$\text{CA}=\frac{TP+TN}{TP+TN+FP+FN}$
AUC	$TPR=\frac{TP}{TP+FN}$*,*$FPR=\frac{FP}{FP+TN}$*,* Then $\text{AUC}=\sum_{i=1}^{n-1}\frac{\left(x_{i+1}-x_{i}\right)\times \left(y_{i}+y_{i+1}\right)}{2}$

## 4 Results and discussion

### 4.1 Extracted advanced features

In the feature extraction process of the acquired vibrational signals for the utilized belt drive systems, the data presented in Fig. 4, Fig. 5 are particularly illuminating. These figures delineate the behavior of the two distinct accelerometers, strategically placed near the driver and driven pulleys, capturing a range of advanced statistical features: Variance, MAD, ZCR, Autocorrelation Coefficient, and Energy of the Signal. These features are analyzed across different operational states, including two RPM levels of 500 RPM and 2000 RPM, applied tensional forces, and conditions (healthy, faulty, and unbalanced). In Fig. 4a and b, the recordings of the first sensor are displayed while in Fig. 4, Fig. 5b, the signals of the second accelerometer are depicted. The variance observed in accelerometer readings is particularly telling. In the healthy operating state, the variance remains comparatively low, indicating a stable and consistent vibrational pattern. However, in faulty and unbalanced states, there is a noticeable increase in variance, suggesting a disruption in the system's usual operational rhythm. This increase can be attributed to irregularities in the belt drive, such as the proposed faults of added weight in the unbalanced state and the mass removal in the faulty state, which introduce additional vibrational components. In addition, MAD is a solid sign of the belt-drive system's anomalies. Moreover, and in any typical operating setting, the average signal intensity is more closely accompanied with the values of MAD. It is also important to point out that some noticeable rises in MAD values are appearing in the faulty and unbalanced states of operation, which is clearly presented in the Y-axis of these mentioned figures in terms of peak values. The more peaks noted, the higher indication of average departure away from the mean value of the signal, and hence, indicating operational irregularities to be detected using the proposed RF model. Interestingly, the frequency components of the vibrational signals are more concerned in the metric of ZCR, as it gives better insights into the signal's spectrum. An elevated ZCR value in the faulty and unbalanced operating conditions indicates a higher frequency rate with which the signal crosses zero, which implies that the system is highly subjectable to unpredictable unnatural behavior. This abnormality must be a response to mechanical damages or faulty states of operation where predictive maintenance takes part. The irregularities of the vibration patterns are resembled by the autocorrelation coefficients, by quantifying the similarity between any signal and its time-delayed analysis. A robust and healthy system is usually characterized by an elevated autocorrelation coefficient, meaning it has consistency predictable pattern of signals. On the contrary, reduced values are an indication of disturbance presence within the system components, which is clearly noted in the operating states of faulty and unbalanced as stated in the Y-axis reduced values. Adding up, the Energy of the signal represents the overall power embedded within the signal itself. In this context, it is exhibiting substantial fluctuations. The higher the operational velocity, where the RPM values increases, the more elevated values of energy within the signal is occurring. In the faulty and unbalanced operational states, it is observed that higher peaks in the energy signal arise, indicating deviations in the proposed belt-drive system which is exercising irregular behavior or system failure. In brief, the examination of these sophisticated statistical characteristics derived from the vibrational signals of belt drive systems provides crucial information regarding the operational condition of the system, as illustrated in Fig. 4, Fig. 5. The fluctuations that have been observed across the operational states establish a strong basis for the development of predictive maintenance strategies. These strategies are designed to identify and prevent faults in belt drive systems at an early stage.

**Fig. 4:** Advance statistical features; Variance, MAD, ZCR, AutoCorrel. Coeff., and Energy of the acquired vibrational signals while operating at 500 RPM: (a) accelerometer 1 readings, where the accelerometer was fixed near the driver pulley; (b) accelerometer 2 recordings, with the sensor positioned next to driven pulley.

**Fig. 5:** Advance statistical features; Variance, MAD, ZCR, AutoCorrel. Coeff., and Energy of the acquired vibrational signals while operating at 2000 RPM: (a) accelerometer 1 readings, where the accelerometer was fixed near the driver pulley; (b) accelerometer 2 recordings, with the sensor positioned next to driven pulley.

Fig. 6 shows a selected case to visualize the novel five vibrational features is presented. When examining the patterns and vibrational behavior, it is seen that the variance and MAD are depicting similar behavior. However, the ZCR and autocorrelation coefficient are of madly fluctuated presentation which suggests a potential lack of diagnostic capability, at least in the current operating state. Furthermore, the energy feature is seen to have the most separating pattern of the three operational states, where the healthy, faulty, and unbalance is clearly seen with the human eye, without the need for diagnostic computer-based capabilities.

**Fig. 6:** Selected operational case of 500 RPM and 150 N belt tension for statistical feature visualization: (a) Variance; (b) MAD; (c) ZCR; (d) Autocorrelation Coeff.; (e) Energy.

Table 5 lists the results from applying the Taguchi method to optimize feature selection for the RF model. The table details the combinations of features tested across eight trials by illustrating the inclusion with number 1 or exclusion with 0. The records the corresponding model accuracy and Signal-to-Noise (S/N) ratios are also give. This systematic approach indicates how different feature combinations impact model performance, as it is clear now that Trial 1 had the highest S/N ratio which suggests an optimal feature set for predictive maintenance.

**Table 5:** Taguchi method results.

Trial	Variance	MAD	ZCR	Autocorrelation Coeff.	Energy	Accuracy (%)	S/N Ratio (dB)
1	1	1	1	1	1	92.0	39.27
2	1	1	0	0	1	89.0	38.99
3	0	1	1	0	1	85.0	38.57
4	0	0	0	1	1	80.0	38.04
5	1	0	1	1	0	88.0	38.88
6	1	0	0	0	0	78.0	37.84
7	0	1	0	1	0	83.0	38.38
8	0	0	1	0	0	75.0	37.50

### 4.2 Tests, scores, and curve analysis

Table 6 enlists the performance and evaluation metrics of the expert system-based RF model which was used in the failure analysis and predictive maintenance strategy for belt drive systems. The table provides a comprehensive overview of the model's efficiency in terms of computational time, data handling capacity, feature input, and predictive accuracy. The model demonstrates remarkable efficiency in terms of computational time, a vital factor in real-time applications. The training phase, requiring only 0.223 s, the testing phase is executed in a mere 0.118 s, showcasing the model's ability to quickly make predictions.

**Table 6:** Efficacy metrics of the deployed Random Forest model.

Model	Train/Test time (Sec.)	Train/Test instances	Total input features	CA	AUC
**Random Forest**	0.223/0.118	80 %/20 %	10 (5 for each accelerometer)	0.990	0.999

For fast and time-effective fault prevention, accurate fault detection is needed in forecasting-based maintenance. Herewith, this time for training and testing the model is highly effective, accurate, and time-friendly. To further analyze the model's performance, it is vital to point out the training and testing portions. 80 percent of the data were trained while the rest were tested with a total number of 100 instances for each case of testing. The input features were 10, 5 for each piezoelectric accelerometer, presented as stated earlier in the advanced feature analysis section. In this analysis, there were no need for important feature selection methods, due to the fact that the total number of features are not exceeding 10 and for the noticed effective time for training and testing the datasets. The CA is noted to be 0.99, as easy as it seems, it was time-consuming to reach this value by try-and-error analysis with different parameters of operation in the RF model until a certain desired CA is reached accordingly. Furthermore, the AUC is called out because the ROC analysis are to be called out later. Interestingly, the AUC has scored a perfect value of 0.999, indicating the model's high dependability in classifying the operational states of the belt-drive system.

To understand whether the parameters of the RF model are efficient, the confusion matrix is called out and depicted in Fig. 7. As stated earlier, for a classification accuracy of 99 %, it is expected to see a confusion matrix with the highest values in the diagonal of the matrix. With a subtotal value of 100 instances for each case, a total value of 1200 is to be predicted based on the trained dataset.

**Fig. 7:** Confusion matrix presentation of the adopted random forest model for all states classification.

The accuracy of the model is clearly reflected in the performance and depiction of the confusion matrix for the twelve utilized cases. For start, it can be clearly seen that when the operating state includes the healthy belts and mechanical system with no added mass imbalances, the highest classification accuracy is induced. That can be explained by the fact that irregularities are hardly detected especially when operating with minimal fault ratios. For instance, when operating it 500 RPM, with a pretensioned belt at 70 N and in a healthy operating status, 100 of the instances are predicted and forecasted correctly as seen in the 500-70-H state of operation. Furthermore, and for further analyzing the confusion matrix, it can also be concluded that faulty and unbalanced operations are marginally fully detected. However, some misclassifications do have fifty percent of the classification right. For instance, the 2000-70-U state instances are predicted as follows: 97 prediction are correct, the remaining 3 are predicted wrong with the majority of them classifying the state as 2000-150-U. the algorithm still gives an indication of unbalance existence, but in a fact that the belt in pretensioned at 150 N instead of 70 N. This is considered a mistake but still a good indication of operational state for future fault prevention of predictive maintenance. This emphasizes the model's versatility in accommodating diverse operational environments. The confusion matrix, reflecting a high degree of accuracy with minimal misclassifications, substantiates the model's suitability in a predictive maintenance context. It adeptly identifies various operational states, particularly faults, thereby enabling proactive maintenance interventions. Adding up to that, Fig. 8 elaborates on the curves of ROC analysis of two randomly selected operating states, namely 500-70-H and 2000-70-H, showcasing the great AOC of 0.999.

**Fig. 8:** ROC analysis curves: (a) 500-70-H operating state; (b) 2000-70-H operating state.

## 5 Conclusion

This study has demonstrated the efficacy of using a Random Forest algorithm for predictive maintenance in belt drive systems, guided by advanced statistical analysis of vibrational data. The key takeaways are.

1. Advanced statistical features, such as Variance, MAD, ZCR, Autocorrelation Coefficient, and Energy of the Signal, have been instrumental in capturing the vibrational characteristics across different operational states which proved to be critical in the analysis, especially when tested by Taguchi method.
2. The expert system's Random Forest model, with its high classification accuracy (CA of 0.990) and AUC (0.999), demonstrated high capability in accurately classifying operational states, including healthy, faulty, and unbalanced conditions.
3. The model's rapid computational performance highlights its suitability for real-time failure and fatigue predictive maintenance applications, a crucial aspect in industrial settings.
4. The robustness of the model is evident in its consistent performance across a variety of operational conditions, including different RPM levels and belt tensions.
5. Insights from the confusion matrix and ROC analysis further substantiated the model's reliability and accuracy while being under challenging operational scenarios.
6. Future work could explore the integration of additional data sources, like temperature or acoustic signals, and the application of other machine learning techniques to enhance predictive accuracy and address more complex fault conditions.
7. Future work can also consider the use of Taguchi method for life prediction assessment and calculation.

## Data availability

The datasets generated in the study are available from the corresponding author on reasonable request.

## CRediT authorship contribution statement

**Ahmed Adnan Shandookh:** Conceptualization, Writing – review & editing. **Ahmed Ali Farhan Ogaili:** Conceptualization, Writing – review & editing. **Luttfi A. Al-Haddad:** Formal analysis, Methodology, Software, Validation, Visualization, Writing – original draft.

## Declaration of competing interest

The authors declare that they have no known competing financial interests or personal relationships that could have appeared to influence the work reported in this paper.
